# Diagnostic Values of Blood Urea Nitrogen (BUN), Creatinine (Cr), and the Ratio of BUN to Cr for Distinguishing Heart Failure from Asthma and Chronic Obstructive Pulmonary Disease

**DOI:** 10.1155/2022/4586458

**Published:** 2022-07-21

**Authors:** Jingjing Zhang, Ling Zhou, Yuezhan Zhang

**Affiliations:** ^1^Department of Nephropathy, Lianyungang TCM Hospital Affiliated to Nanjing University of Chinese Medicine, Lianyungang, Jiangsu 222000, China; ^2^Department of Emergency, Lianyungang TCM Hospital Affiliated to Nanjing University of Chinese Medicine, Lianyungang, Jiangsu 222000, China; ^3^Department of Geriatrics, Lianyungang TCM Hospital Affiliated to Nanjing University of Chinese Medicine, Lianyungang, Jiangsu 222000, China

## Abstract

**Background:**

In clinical practise, it can be challenging to tell the difference between asthma and chronic obstructive pulmonary disease (COPD) and heart failure (HF), which share comparable dyspnea symptoms. We aimed to examine whether renal function indexes blood urea nitrogen (BUN), creatinine (Cr), and the ratio of BUN to Cr (BUN/Cr) can be used to distinguish HF from asthma and COPD.

**Methods:**

A total of 170 patients were admitted for dyspnea symptoms in this retrospective study. There are 69 patients with HF (HF group), 50 patients with asthma (asthma group), and 51 patients diagnosed with COPD (COPD group). The levels of BUN, Cr, and the ratio of BUN/Cr in the three groups were compared. Student's *t*-test or the one-way analysis of variance (ANOVA) test was used to compare means. Using the area under the receiver operating characteristic curve, model differentiation was evaluated (AUC). *Z*-test comparisons of AUC were carried out.

**Results:**

Compared with the asthma/COPD group (asthma group + COPD group) or the COPD group, the levels of BUN and Cr were raised in the HF group, while there was no significant difference of the BUN/Cr ratio. Compared with those in the asthma group, the levels of BUN, Cr, and BUN/Cr ratio were significantly increased in the HF group (all *p* < 0.05), whereas no significant differences of BUN, Cr, and BUN/Cr ratio were found between asthma and COPD. The AUC in distinguishing HF from asthma/COPD were 0.736 and 0.751 for BUN and Cr, respectively, and no significant difference was observed between BUN and Cr. The cutoff values (specificity, sensitivity, and Youden index) in distinguishing between HF and asthma/COPD were 20.45 mg/dL (79.21%, 56.52%, and 0.357) for BUN and 0.782 mg/dL (72.28%, 68.12%, and 0.404) for Cr, respectively.

**Conclusions:**

BUN and Cr showed accurate and reliable diagnostic values which could be potential biomarkers for differentiating HF from asthma and/or COPD.

## 1. Introduction

Dyspnea, due to its high prevalence [1], was among the top ten principal reasons for adult presentation to the emergency department (ED) [2, 3]. There are a number of conditions that can lead to dyspnea, including heart failure (HF), asthma, and chronic obstructive pulmonary disease (COPD). HF is a condition in which the heart cannot pump enough blood efficiently, while asthma and COPD are associated with chronic airway inflammation. A common sign of cardiopulmonary disease, dyspnea can range from moderate and short lived to severe and persistent. In clinical practise, it can be challenging to distinguish between HF, asthma, and COPD because they all have comparable dyspnea symptoms. At this point, the right diagnostic laboratory tests may be beneficial to support a particular diagnosis and so play a vital role in justifying a more rapid evaluation and precise therapies.

Brain natriuretic peptide (BNP) [4, 5] and N-terminal pro-B-type natriuretic peptide (NT-proBNP) [6, 7], as recommended by guidelines, are valuable tools in distinguishing HF from asthma/COPD. However, this multitude of causes for the elevation of BNP or NT-proBNP, such as age and renal insufficiency, imposes limits on its diagnostic use for HF [4]. Furthermore, the measurement of BNP or NT-proBNP is expensive and increases the economic burden of patients. Thus, whether there are other common and cheap emergency blood tests that can help distinguish HF from asthma/COPD remains a challenging issue concerned by clinicians, when they encounter patients with dyspnea attack.

Aronson et al. [8] investigated 541 patients with decompensated HF and found that the blood urea nitrogen (BUN) and BUN/creatinine (BUN/Cr) ratio, but not serum Cr, remained related to mortality after adjusting for other risk factors during the follow-up period. Another study done by Filippatos et al. [9] came to a similar conclusion: after controlling for covariates, BUN, but not Cr, is a statistically significant predictor of mortality and the composite endpoint of death or heart failure hospitalization at 60 days after discharge. Georgiopoulou et al. [10] revealed that serum Cr in outpatients with HF was an adequate prognosticator of death or HF hospitalization and elevated BUN was associated with well all-cause and cardiovascular hospitalization rates and ED visits rates. Parrinello et al. [11] found that higher values of BUN in HF with a preserved ejection fraction was related to significantly increased all-cause mortality. Up to now, it remains uncertain whether these cheap and easy-to-obtain renal function indices (BUN, Cr, and BUN/Cr ratio) could differentiate HF from asthma/COPD preliminarily. To the best of our knowledge, there has not yet been a discussion on how to compare the diagnostic values of these renal function indicators to differentiate between HF and asthma/COPD. Our study may provide novel evidence for whether BUN, Cr, and BUN/Cr ratio could demonstrate accurate and reliable diagnostic values in distinguishing HF from asthma/COPD.

The paper's organization paragraph is as follows: the materials and methods is presented in Section 2.  Section 3 discusses the experiments and results.  Section 4 consists of the discussion section. Finally, in Section 5, the research work is concluded.

## 2. Materials and Methods

### 2.1. Study Population

A total of 170 patients with dyspnea attack admitted to Lianyungang TCM Hospital Affiliated to Nanjing University of Chinese Medicine were consecutively enrolled in this study between January 2018 and February 2021. The diagnoses of HF, asthma, and COPD were performed following the relevant guidelines [12–14]. All patients underwent echocardiography, pulmonary function test, electrocardiography, chest computed tomography, and BNP or NT-proBNP if necessary, except for cases with HF or asthma/COPD confirmed by other hospitals recently. Finally, a total of 69 inpatients were diagnosed with HF (HF group) and the rest were inpatients with asthma or COPD (asthma group 50; COPD group 51). Inclusion criteria were adults ≥ 30 years old, at least symptoms presenting at the time of visit, and emergency renal function tests in the ED or on admission performed by all patients. Patients with comorbidities between HF, asthma, and COPD, patients who underwent renal function tests on the second day after admission, patients whose clinical data were incomplete, patients with gastrointestinal bleeding, kidney disease, thyroid disease, shock, trauma, pregnant women, and patients with other causes of dyspnea were all excluded. The study followed the *Declaration of Helsinki* and was approved by the ethics committee of Lianyungang TCM Hospital Affiliated to Nanjing University of Chinese Medicine.

### 2.2. Clinical Data

Medical records of patients admitted to Lianyungang TCM Hospital Affiliated to Nanjing University of Chinese Medicine were used to compile baseline data. The Hitachi7600 automatic biochemical analyzer was used to determine renal function variables (BUN and Cr). The BUN/Cr ratio was calculated and recorded (BUN: 1 mg/dL = 0.357 mmol/L, Cr: 1 mg/dL = 88.4 *μ*mol/L).

### 2.3. Statistical Analysis

Statistical analysis was performed using SPSS v19.0 (SPSS, Chicago, USA). Descriptive analysis of continuous variables was used to calculate the mean and standard deviation. Qualitative data were compared using the chi-squares test. Means were compared using Student's *t*-test or one-way analysis of variance (ANOVA) test for independent samples. Prognostic performance was tested by calculating receiver operating characteristic (ROC) curves and displayed in AUC. Comparison of AUC was performed using the *Z*-test of the software MedCalc v18.2.1 (MedCalc, Ostend, Belgium). From the ROC coordinates, the score value with the best Youden index (sensitivity + specificity − 1) was used to determine the cutoff value for the above scores. *p* < 0.05 was considered statistically significant.

## 3. Results

### 3.1. Patients' Characteristics

A total of 69 inpatients diagnosed with HF (HF group) and 101 cases with asthma and COPD (asthma group 50; COPD group 51) were analyzed. The mean age of the study sample was 73.12 ± 12.12 years. Among them, 103 (60.6%) were female and 67 (39.4%) were male. There were no significant differences of age or the rate of coronary heart disease (all *p* > 0.05), except for the rates of gender, diabetes mellitus, and hypertension between HF and asthma/COPD (Table 1) and among three groups of HF, asthma, and COPD (Table 2). Renal function indices were the focus of the present study.

### 3.2. BUN, Cr, and the BUN/Cr Ratio

As shown in Table 1 and Figures 1(a)–1(c), the levels of BUN and Cr were boosted in the HF group compared with the asthma/COPD group (asthma group + COPD group) (all *p* < 0.05), BUN and Cr levels were higher in the HF group compared to the COPD group following pairwise comparison of subgroup analysis, but the BUN/Cr ratio did not differ (*p* > 0.05) (all *p* < 0.05), while there was no difference in the BUN/Cr ratio (*p* > 0.05) (T2, Figures 2(a)–2(c)); furthermore, the levels of BUN, Cr, and BUN/Cr ratio were promoted in the HF group compared with the asthma group (all *p* < 0.05), whereas no differences of BUN, Cr, and BUN/Cr ratio were found between asthma and COPD (all *p* > 0.05).

### 3.3. Comparison of ROC Curves of BUN, Cr, and BUN/Cr Ratio in Distinguishing Different Groups

The AUC (95% confidence interval (CI)) in distinguishing between HF and asthma/COPD were 0.736 (0.663 to 0.800) for BUN and 0.751 (0.679 to 0.814) for Cr (Figure 3). The cutoff values (specificity, sensitivity, and Youden index) in distinguishing between HF and Asthma/COPD were 20.45 mg/dL (79.21%, 56.52%, and 0.357, respectively) for BUN and 0.782 mg/dL (72.28%, 68.12%, and 0.404, respectively) for Cr. One result of subgroup analysis was that the AUC (95% (CI)) in distinguishing between HF and asthma were 0.760 (0.673 to 0.834) for BUN, 0.726 (0.636 to 0.804) for Cr, and 0.621 (0.528 to 0.708) for BUN/Cr ratio (Figure 4). The cutoff values (specificity, sensitivity, and Youden index) in distinguishing between HF and asthma were 19.86 mg/dL (82.00%, 59.42%, and 0.414, respectively) for BUN, 0.842 mg/dL (76.00%, 62.32%, and 0.383, respectively) for Cr, and 21.26 (50.00%, 69.57%, and 0.196, respectively) for the BUN/Cr ratio. The other result of subgroup analysis was that the AUC (95% (CI)) in distinguishing between HF and COPD were 0.712 (0.622 to 0.791) for BUN and 0.776 (0.691 to 0.847) for Cr (Figure 5). The cutoff values (specificity, sensitivity, and Youden index) in distinguishing between HF and COPD were 20.45 mg/dL (76.47%, 56.52%, and 0.330, respectively) for BUN and 0.782 mg/dL (78.43%, 68.12%, and 0.466, respectively) for Cr.

## 4. Discussion

HF, asthma, and COPD are the most common and important differential diagnoses for dyspnea in older adults. Despite the three diseases' fundamentally different pathophysiology, their comparable clinical presentations make it challenging for clinicians to make a diagnosis and assess the severity of the underlying condition [6]. What is worse, overlapping clinical presentations (e.g., asthma and COPD) and comorbid diseases (e.g., HF and COPD) can conspire to confound accurate diagnosis and optimal therapy [15].Thus, rapid evaluation and targeted diagnostic studies are of central importance for reducing mortality and disease burden [16].

In the present study, we have proved that BUN was raised in the HF group compared with the asthma/COPD group (*p* < 0.001), suggesting that BUN could be used to distinguish between HF and asthma/COPD. Furthermore, after pairwise comparison of subgroup analysis, BUN was elevated in the HF group compared with the asthma or COPD group (all *p* < 0.001), suggesting that BUN could be used to distinguish not only between HF and asthma but also between HF and COPD, similarly. However, there was no significantly statistical difference of BUN between asthma and COPD, indicating that BUN could not be used to distinguish them.

Next, Cr has also been found to show the same trend, suggesting that Cr could be applied to distinguish HF from asthma/COPD (*p* < 0.001). Additionally, following pairwise comparison of the subgroup analysis, Cr could be used to similarly distinguish between HF and COPD as well as between HF and asthma (all *p* > 0.001). However, Cr could not be applied to differentiate asthma from COPD (*p* > 0.05).

Moreover, with respect to the BUN/Cr ratio, we proved that no significant difference was observed between HF and asthma/COPD, suggesting that the BUN/Cr ratio could not be used to distinguish HF from asthma/COPD (*p* > 0.05). After pairwise comparison of subgroup analysis, the BUN/Cr ratio could not be used to distinguish between COPD and HF or asthma (*p* > 0.05), similarly. However, the BUN/Cr ratio could be used to differentiate HF from asthma (*p* > 0.05).

Finally, we also discovered that the AUC in distinguishing between HF and asthma/COPD were 0.736 for BUN and 0.751 for Cr and no significant difference was observed between BUN and Cr (*Z* = 0.389, *p* = 0.697) (Figure 3). Subgroup analysis showed that the AUC in distinguishing between HF and asthma were 0.760 for BUN, 0.726 for Cr, and 0.621 for the BUN/Cr ratio and the only significant difference was observed between BUN and the BUN/Cr ratio (0.760 vs. 0.726, *Z* = 0.736, *p* = 0.462; 0.760 vs. 0.621, *Z* = 3.063, *p* = 0.002; and 0.726 vs. 0.621, *Z* = 1.299, *p* = 0.194) (Figure 4). In other words, BUN could demonstrate better performance in distinguishing between HF and asthma than the BUN/Cr ratio. The other result of subgroup analysis was that the AUC in distinguishing between HF and COPD were 0.712 for BUN and 0.776 for Cr and no significant difference was observed between BUN and Cr (*Z* = 1.337, *p* = 0.181) (Figure 5).

We hypothesised that the causes of the aforementioned aberrant renal function indices in HF may be related to neurohormonal activation in addition to renal hypoperfusion brought on by abrupt hemodynamic changes during bouts of decompensation [8, 10, 17]. In addition, we have found that there were significantly statistical differences of the rates of diabetes mellitus and hypertension in the HF group compared with the asthma and/or COPD group (*p* < 0.05), suggesting that the common comorbidities (diabetes mellitus and hypertension) of HF could lead to the adverse effects on renal function [18]. Fedeli et al. [19] proved that renal dysfunction in COPD patients might be associated with systemic inflammation and malnutrition. Asthma kidney dysfunction may be caused by behavioural or biological variables such inactivity and inflammation, according to research by Huang et al. The reason for the differences of renal function indices among HF, asthma, and COPD might be related to the abovementioned mechanisms.

We are aware of this study's shortcomings. First off, since this was a retroactive examination, a more exacting design was omitted. Second, from a single-center perspective, the sample size is small. Third, there is heterogeneity in the sample (e.g., different onset-to-admission intervals, different disease severity, and different comorbidity ratios). To validate findings, larger, more homogeneous samples from multicenter research are required.

## 5. Conclusion

BUN and Cr exerted accurate and reliable diagnostic value, suggesting that they were potential biomarkers for differentiating HF from asthma and/or COPD.

## Figures and Tables

**Figure 1:** Comparison of BUN (a), Cr (b), and BUN/Cr ratio (c) between HF and asthma/COPD. HF: heart failure; COPD: chronic obstructive pulmonary disease; BUN: blood urea nitrogen; Cr: creatinine; BUN/Cr ratio: BUN to Cr ratio; ^∗∗∗^*p* < 0.001.

**Figure 2:** Comparison of BUN (a), Cr (b), and BUN/Cr ratio (c) among HF, asthma, and COPD. HF: heart failure; COPD: chronic obstructive pulmonary disease; BUN: blood urea nitrogen; Cr: creatinine; BUN/Cr ratio: BUN to Cr ratio; ^∗^*p* < 0.05, ^∗∗∗^*p* < 0.001.

**Figure 3:** Comparison of ROC curves of BUN and Cr in distinguishing HF from asthma/COPD. HF: heart failure; COPD: chronic obstructive pulmonary disease; BUN: blood urea nitrogen; Cr: creatinine.

**Figure 4:** Comparison of ROC curves of BUN, Cr, and BUN/Cr ratio in distinguishing HF from asthma. HF: heart failure; BUN: blood urea nitrogen; Cr: creatinine; BUN/Cr ratio: blood urea nitrogen to creatinine ratio.

**Figure 5:** Comparison of ROC curves of BUN and Cr in distinguishing HF from COPD. HF: heart failure; COPD: chronic obstructive pulmonary disease; BUN: blood urea nitrogen; Cr: creatinine.

**Table 1:** Comparison of the levels of different variables between two groups.

Variables	HF group (*n* = 69)	Asthma/COPD group (*n* = 101)	*p* value
Age (years)	72.25 ± 14.54	73.71 ± 10.19	0.470
Gender (male/female)	40/29	27/74	<0001^∗^
Hypertension (Y/N)	44/25	42/69	0.001^∗^
Diabetes mellitus (Y/N)	23/46	16/85	0.008^∗^
Coronary heart disease (Y/N)	22/47	22/79	0.140^∗^
BUN (mg/dL)	24.41 ± 10.90	16.46 ± 5.58	<0.001
Cr (mg/dL)	0.98 ± 0.37	0.73 ± 0.23	<0.001
BUN/Cr ratio	25.66 ± 8.70	23.43 ± 7.97	0.087

Quantitative data were present as mean ± standard deviations; Y: yes; N: no; HF: heart failure; COPD: chronic obstructive pulmonary disease; BUN: blood urea nitrogen; Cr: creatinine; BUN/Cr ratio: BUN to Cr ratio; ^∗^Student's *t*-test or chi-squared test.

**Table 2:** Comparison of the levels of different variables among three groups.

Variables	HF group (*n* = 69)	Asthma group (*n* = 50)	COPD group (*n* = 51)	*p* value
Age (years)	72.25 ± 14.54	72.08 ± 11.11	75.31 ± 9.02	0.304
Gender (male/female)	40/29	13/37	14/37	<0001^∗^
Hypertension (Y/N)	44/25	24/26	17/34	0.004^∗^
Diabetes mellitus (Y/N)	23/46	8/42	8/43	0.029^∗^
Coronary heart disease (Y/N)	22/47	13/37	9/42	0.212^∗^
BUN (mg/dL)	24.41 ± 10.90	15.82 ± 5.31	17.10 ± 5.82	<0.001
Cr (mg/dL)	0.98 ± 0.37	0.75 ± 0.24	0.71 ± 0.23	<0.001
BUN/Cr ratio	25.66 ± 8.70	21.86 ± 6.64	24.98 ± 8.87	0.039

Quantitative data were present as mean ± standard deviations; Y: yes; N: no; HF: heart failure; COPD: chronic obstructive pulmonary disease; BUN: blood urea nitrogen; Cr: creatinine; BUN/Cr ratio: BUN to Cr ratio; ^∗^ANOVA test or chi-squared test.

## Data Availability

All data generated or analyzed during this study are included in this published article.
